RETRACTED

# Research and Application of the Data Mining Technology in Economic Intelligence System

**DOI:** 10.1155/2022/6439315

**Published:** 2022-03-15

**Authors:** Qingqing Chang, Jincheng Hu

**Affiliations:** School of Information Management, Shanghai Lixin University of Accounting and Finance, Shanghai 201209, China

## Abstract

In the context of the rapid development of the modern economy, information is particularly important in the economic field, and information determines the decision-making of enterprises. Therefore, how to quickly dig out information that is beneficial to the enterprise has become a crucial issue. This topic applies data mining technology to economic intelligent systems and obtains the data object model of economic intelligent systems through the integration of information. This article analyzes the interrelationship between its objects on this basis and uses data mining-related methods to mine it. The establishment of economic intelligence systems not only involves the establishment of mathematical models of economic systems, but also includes research on the algorithms applied to them. How to apply an algorithm to quickly and accurately extract the required economic intelligence domain information from the potential information in the database, or to provide a method to find the best solution, involves the use of association rules and classification prediction methods. The application of data mining algorithms can be used to study the application of economic intelligence systems. This paper develops and designs an economic intelligence information database and realizes the economic intelligence system on this basis, and realizes the research results. Finally, this paper has tested the dataset, and the results show that the classification accuracy of this algorithm is 2.64% higher than that of the ID3 algorithm.

## 1. Introduction

Following the Internet, digital mining has become a new research hotspot, especially in high-dimensional, large-scale, distributed digital mining, which has broader prospects, and the potential economic value is also limitless. Among them, the classification prediction technology will assist future smart business activities and provide important reference decisions.

Regarding the data mining technology and economic intelligence systems, scholars at home and abroad have provided a lot of references. Li and Long studied image detection and quantitative detection analysis of gastrointestinal diseases based on data mining [1]. Zuo researched and analyzed the characteristics of network viruses and designed a computer data mining module. He combined the data mining technology with the dynamic behavior interception technology to mine hidden information and determine whether there is a virus. He applied this method to network Trojan virus detection [2]. Buczak and Guven provide a short tutorial description of machine learning (ML) methods and data mining (DM) methods for network analysis [3]. Xu et al. look at privacy issues related to data mining from a broader perspective and study various methods that help protect sensitive information. He reviewed the most advanced methods and put forward some preliminary ideas for future research directions [4]. Yan and Zheng found that even after considering data mining, many fundamental signals are important predictors of cross-sectional stock returns. Yan and Zheng's method is universal, and Yan and Zheng also applied it to past returns-based anomalies [5]. Emoto et al. use terminal restriction fragment length polymorphism (T-RFLP) data mining analysis to elucidate the gut microbiota profile of patients with coronary artery disease [6]. Hong et al. proposed a new method to construct a flood sensitivity map in Poyang County, Jiangxi Province, China, by implementing the fuzzy Wolfe and data mining methods [7]. The data results of these studies are not comprehensive, and the results lack basis; thus, they cannot be recognized by the public.

RETRACTED

The innovative point of this research on the realization of economic intelligence systems based on the data mining technology lies in the use of a combination of association rules and clustering two data mining methods to realize data information mining. It can not only mine the potential information of the data well, but also improve the efficiency of data mining. This research uses the least mean square algorithm to optimize the research, which improves the experimental effect to a certain extent.

## 2. Data Mining Technology and Economic Intelligence Systems

### 2.1. Data Warehouse

#### 2.1.1. The Concept of Data Warehouse

A data warehouse is a subject-oriented, integrated, irreplaceable, and time-changing collection used to support the analysis, decision-making, and development of an enterprise or organization. The data warehouse is a powerful combination of different resources. After integration, it will change according to the theme and contain historical data, and the data stored in the archive are usually no longer edited [8, 9].

The theme is the abstract concept of integrating, categorizing, analyzing, and using information in high-level organizational information systems [10]. Logically speaking, this is consistent with the analysis goals related to the subject's macro-analysis field. Themes benefit from a series of tables in the database. Themes can be stored in a multidimensional database. The division of themes must ensure the independence of each theme. Data warehouse integration is the process of extracting, filtering, cleaning, and merging distributed data to meet the needs of decision analysis, to integrate the data in the database [11].

RETRACTED

#### 2.1.2. The Architecture of the Data Warehouse

Simply put, a data warehouse consists of operable external data sources, one or more databases, and one or more data analysis tools. Therefore, its realization process should include three major steps: collecting various source data, storing and managing data, and obtaining the required information. The architecture of the data warehouse is shown in Figure 1.

The data processing flow of the data warehouse is as follows:

1. Take out the data needed for decision-making from any business processing system source[12];
2. Clean up and integrate data sources;
3. Load and update the data warehouse according to the theme [13]; the loading is to load metadata. The basic framework and the description of the metadata management system are shown in Figure 2.
4. According to the needs of the decision support system, organize the data and information in various forms [14];
5. Decision-making, data analysis, and processing capabilities and data mining;
6. Flexible and diverse results expression.

In the field of data warehouse, metadata is divided into technical metadata and business metadata according to usage. First, metadata can provide user-based information. For example, metadata that records business description information of data items can help users use data. Secondly, metadata can support the management and maintenance of data in the system. For example, metadata about the storage method of data items can support the system to access data in the most effective way.

#### 2.1.3. OLAP Technology

Online analysis and processing technology was proposed in 1993 by the inventor of relational data. This technology gives the concept of online analysis of data and has good effects on multidimensional information processing. It has developed rapidly in recent years [15]. Online analytical processing is to enable analysts, managers, or executives to quickly, consistently, and interactively access information from multiple perspectives. This information is transformed from the original data, can be truly understood by users, and truly reflects the situation of the enterprise. It is a type of software technology that achieves a deeper understanding of data. The technical framework diagram of the OLAP engine is shown in Figure 3.

OLAP can be divided into categories according to different data composition methods: relational OLAP, multidimensional OLAP, and hybrid OLAP [16, 17].

RETRACTED

The following briefly introduces the core organization model of the OLAP technology:

  Relational online analytical processing (ROLAP, Relational OLAP): This method is mainly used for the processing and analysis of relational databases, and the organization of data usually adopts a snowflake-shaped method [18].
  Multidimensional online analytical processing (MOLAP, Multi-Pimensicnal, OLAP): This method relies on indexing technology; first, it preprocesses the advanced nature of the relational data, organizes it into the form of multidimensional data, analyzes and builds indexes, and performs retrieval [19].
  Front-end online analysis (Desktop OLAP): It is a data analysis method that partially downloads data from the server to the client and can reorganize the data on the client. It provides flexible and simple information processing [20]. The difference between online analytical processing and online transaction processing is shown in Table 1.

### 2.2. Technical Basis of Data Mining

#### 2.2.1. Concepts and Characteristics of Data Mining

Data mining is a series of methods and techniques used to extract knowledge from data. The extraction process is very complicated, mainly due to the large-scale, irregular, and noisy characteristics of the data [21].

The general process of knowledge discovery is as follows:

1. Identify and gradually understand the application areas.
2. Select the dataset to be studied.
3. Data integration.
4. Data cleaning, deduplication, and error removal.
5. Develop models and construct hypotheses.
6. Data mining.
7. Interpret and express the results and display them in a humane way.
8. Inspection results.
9. Manage the discovered knowledge.

Data mining technology has the following characteristics:

1. The amount of data is often very large [22, 23]. The so-called data mining must be built on the basis of massive data, as small-scale data cannot reflect statistical laws. It is completely meaningless to mine small-scale data, and the knowledge found is not enough to reflect the actual situation in real life. It can be said that it is essentially wrong. In the face of massive amounts of data, it is particularly important to reduce the time complexity of the related algorithms, so that real useful knowledge and information can be mined in an effective time.
2. Potentially useful [24]: The result of data mining should be an undiscovered rule or pattern, which can provide certain guidance for life and production. The results of excavations like “Many people holding umbrellas on rainy days” are meaningless.
3. Independence and indivisibility: The data mining process is an extremely complex process, which cannot be completed in a few simple steps. However, these steps cooperate with each other and cannot complete the corresponding work independently. In this process, on the one hand, it is necessary to select specific algorithms to achieve efficiency of mining, and on the other hand, the relevant operators are required to have solid business skills. It can analyze and process data according to actual business needs, make reasonable interpretations of the mining results, and correctly apply them to future actual work.

RETRACTED

#### 2.2.2. Methods of Data Mining

Data mining methods can be divided into descriptive analysis and predictive analysis according to their realized functions. In the final analysis, descriptive analysis is a useful preparation for predictive analysis. It fully reflects the overall distribution of the data and can show the inherent characteristics of the relevant data. Correspondingly, predictive analysis is based on descriptive analysis and treats its analysis results from a developmental perspective, thereby generating a prediction of future data. It gives the final decision-maker a data-level reminder. Predictive analysis mainly refers to prediction based on classification or based on statistical regression problems. At the same time, the main representatives of descriptive analysis are association rule mining and cluster analysis methods. Several common methods of classification, clustering, and association rules are introduced.

*(1) Classification*. Classification is the process of categorizing data into different categories based on a well-defined conceptual description. The naive Bayes method of statistics and the decision tree learning method in machine learning are the different implementations of classification techniques.

*(2) Association Rules*. The core purpose of the association rule analysis is to discover the interrelated and interdependent relationships that exist in the data. Association rule mining is also a data mining method derived from database theory. Specifically, in relational databases, there are often some data that appear synchronously, which is called a pattern. When this pattern appears frequently in the database, it is considered that there is a specific association relationship, which is called an association rule. It is determined that the revised content is consistent with the original intention of the author. The current research generally uses support and confidence as its measurement criteria. In the research process, scholars further strengthened the relevant parameters of association rules from different perspectives. It incorporates the interest level and other indicators into the consideration range; thus, many new methods and new applications have been proposed, and new developments in association rule mining have also appeared.

RETRACTED

When specific patterns in the dataset meet the support and confidence thresholds, they become the association rules contained in it. First, the mining results need to reflect the closeness of the connections between the data. Data with less connections should not appear as a result of the association rules. Therefore, a reasonable minimum support threshold needs to be set. At the same time, we also pay attention to the credibility of the association rules and make reasonable requirements for the credibility, which is reflected in the setting of the minimum confidence threshold. For example, assuming that the minimum support rate is 50% and the minimum confidence rate is 50%, then *A*⇒*C*. Details are shown in Table 2.

*(3) Clustering*. Compared with association rules, cluster analysis is another common method of data mining. It refers to a certain similarity estimation of the data to be analyzed in an unsupervised environment, and the data with higher similarity is combined, which is called clustering. The clustered result set has the characteristics of similarity of the same class and differences between classes, which is very suitable for grasping the distribution of data and its association.

*(4) Sequence*. Sequence pattern analysis is similar to association analysis, and its purpose is to dig out the connections between data, but the focus of sequence pattern analysis is to analyze the causal relationship between the data before and after.

#### 2.2.3. The Architecture of Data Mining

The core technology of DM is artificial intelligence, machine learning, statistics, etc., but a DM system is not a simple combination of multiple technologies, but a complete whole. It also needs the support of other assistive technologies to complete a series of tasks of data collection, preprocessing, data analysis, and result presentation, and finally present the analysis results to the user. According to the functions, the entire data mining system can be roughly divided into a three-level structure, as shown in Figure 4.

#### 2.2.4. The Steps of Data Mining

The four steps of data mining can be summarized as follows:

1. Data selection
2. Data transformation
3. Mining data
4. Interpret the results

The completion of the data selection process obtains the specific partial data needed for data mining. At this time, it is necessary to further format the selected data to provide an identifiable data input source for the next step of data mining.

After the completion of the two tasks of data selection and data format conversion, the next step is to use various data mining algorithms and integrated tools for the mining process. In the mining process, data warehouse and data mining algorithms are often used in combination. On the one hand, it reduces the calculation of specific statistical values; on the other hand, it reduces the consumption of extra time and space resources generated by data exchange. Although this is a commonly used method, it does not actually restrict the algorithm from using the original data under appropriate conditions. In most cases, this approach is essential. The main advantage of using a data warehouse is that most of the data has been integrated into a suitable format, making it easier for data mining tools to extract high-quality information.

RETRACTED

A reasonable interpretation of the mining results is the final step in the process. Through the steps, the mining results after analysis and processing are obtained. In this step, these mining results need to be sent to the final decision-maker through the DSS. Interpreting the mining results not only requires a reasonable interpretation of the results itself, but also requires a deeper filtering of the data before sending it to the decision-making system. Once the mining results are unexplainable or unsatisfactory, the entire mining process needs to be repeated until useful results are produced.

In summary, data mining is not only an independent and indivisible process, but the realization of the process is also extremely complicated. Before data can be provided to data mining tools, many steps need to be performed correctly. In addition, we cannot guarantee that the existing data mining tools will not produce meaningless results during the work process. Here, to a large extent, data mining is not a direct analysis operation on the original data, but is based on a data warehouse, and the data warehouse provides a direct source of input data to the data mining tool. At the same time, the DSS tool will make the next step of processing the mining results. In this way, data mining will be combined with DSS to provide a final solution for enterprises to implement data mining strategies. In general, the developers of data mining tools are also the people who preprocess the data. Therefore, a well-designed data mining tool will integrate related tools for data integration and format conversion. It is worth noting that although data mining uses data warehouses to provide processed data as input, in most cases, it is not necessary. Data can be downloaded directly from the operation file to a general file, which contains data that can be used for data mining and analysis.

Data mining technologies will deepen the economic statistics accumulated over a long period of time into the conditions required by data users. Many characteristics of the data mining technology will be involved in the process of practice. According to these characteristics, ensure that economic statistics can play a role to the greatest extent and serve the needs of managers.

RETRACTED

### 2.3. Economic Intelligence Systems

Economic data mining is the introduction of data mining methods and techniques in computer technology into economic research, and the integration of data mining and econometric methods. It has interdisciplinary characteristics. The problems caused by information technology often push the technology forward. The large amount of historical data accumulated by the database system provides data support and technical background for data mining and has a wide range of applications.

First, it creates an economic data warehouse and an economic data mining model. It includes a collection of economic indicator data, the establishment of a data warehouse, the cleaning, conversion, loading, and drilling of data, and the selection of economic data mining models. Then, it conducts data analysis through the model, performs multidimensional OLAP analysis and data display, and performs methods such as association, clustering, and abnormal data analysis. By observing measurement results, analyzing economic phenomena, predicting possible situations, and discovering knowledge, it provides a basis for scientific decision-making and obtains valuable information from it. Finally, it is applied to management decision-making and becomes an auxiliary tool for related departments or enterprises. The basic framework of OLAP modeling is shown in Figure 5.

In the application of economic data mining technology, enterprise managers can be used for data warehouse creation, data loading, and drilling. The update of multidimensional datasets uses analysis managers to establish fact tables, dimensions, and granularity. Through the creation of multidimensional datasets, OLAP is realized, and economic data mining models are selected to conduct data mining. The basic framework and description of the OLAP analysis service are shown in Figure 6.

The development environment of the economic intelligence system is shown in Table 3.

## 3. The Least Mean Square Algorithm

The weight vector *ϖ* is defined using the least mean square algorithm (LMS) learning rule:

(1) $$\begin{array}{c} \varpi_{n+1}=\varpi_{n}+\Delta \varpi_{n}\\ =\varpi_{n}-{\eta \frac{\partial P}{\partial \overset{-}{W}}|}_{n}, \end{array}$$

(2) $$\begin{array}{c} \beta =\varpi^{T}a, \end{array}$$

(3) $$\begin{array}{c} \phi =f\left(\beta \right)\\ =f\left(\varpi^{T}a\right), \end{array}$$

(4) $$\begin{array}{c} \varsigma =\lambda -\phi \\ =\lambda -\left(\varpi^{T}a\right). \end{array}$$

The formula of the cost function *P* is as follows:

(5) $$\begin{array}{c} P=\frac{1}{2}\varsigma^{2}\\ =P\left(\varpi \right). \end{array}$$

*P* takes the partial derivative of each element of *ϖ*, namely,

(6) $$\begin{array}{c} \nabla P\left(\varpi \right)=\frac{\partial P}{\partial \beta }\frac{\partial \beta }{\partial \varpi }. \end{array}$$

Applying the chain rule through formula (6), we get

(7) $$\begin{array}{c} \nabla P\left(\varpi \right)=\frac{\partial P}{\partial \varsigma }\frac{\partial \varsigma }{\partial \phi }\frac{\partial \phi }{\partial \beta }\frac{\partial \beta }{\partial \varpi }. \end{array}$$

Differentiate *ς* on both sides of formula (5), and we have

(8) $$\begin{array}{c} \frac{\partial P}{\partial \varsigma }=\varsigma . \end{array}$$

At the same time, formula (4) is differentiated on both sides of *ϕ*, and there are

(9) $$\begin{array}{c} \frac{\partial P}{\partial \varsigma }=-1. \end{array}$$

At the same time, formula (3) is differentiated on both sides of *β*, and there are

(10) $$\begin{array}{c} \frac{\partial \phi }{\partial \beta }=f^{\prime }\left(\beta \right). \end{array}$$

Finally, formula (2) is differentiated on both sides of *ϖ*, and there are

(11) $$\begin{array}{c} \frac{\partial \beta }{\partial \varpi }=a. \end{array}$$

Incorporating formula (11) into formula (7), we get

(12) $$\begin{array}{c} \nabla P\left(\varpi \right)=-\varsigma f^{\prime }\left(\beta \right)a. \end{array}$$

Therefore, when *n* is presented in the network, the LMS learning rule can be written as

(13) $$\begin{array}{c} \varpi_{n+1}=\varpi_{n}+\Delta \varpi_{n}\\ =\varpi_{n}-\eta \nabla E\left(\varpi_{n}\right)\\ =\varpi_{n}+\eta \varsigma f^{\prime }{\left(\beta \right)}_{n}a_{n}. \end{array}$$

Formulate the error signal term *ψ* for the output layer:

(14) $$\begin{array}{c} \lambda =\varsigma f^{\prime }\left(\beta \right)\\ =\left(\lambda -\phi \right)f^{\prime }\left(\beta \right). \end{array}$$

Therefore, formula (13) can be written as

(15) $$\begin{array}{c} \varpi_{n+1}=\varpi_{n}+\Delta \varpi_{n}\\ =\varpi_{n}+\eta \psi_{n}a_{n}. \end{array}$$

For mode *n*, formula (13) can be written as the form *ϖ*_*m*,*n*_ of each vector component of the weight vector *ϖ*_*n*_:

(16) $$\begin{array}{c} \varpi_{n+1}=\varpi_{n}+\eta \left(\lambda_{n}-\phi_{n}\right),\\ f^{\prime }\left(\beta \right)a_{m,n}=\varpi_{m,n}+\eta \psi_{n}a_{m,n}. \end{array}$$

The error signal is equal to the error:

(17) $$\begin{array}{c} \lambda =\varsigma f^{\prime }\left(\beta \right)\\ =\varsigma \\ =\lambda -\phi ,\\ \varpi_{n+1}=\varpi_{n}+\Delta \varpi_{n}\\ =\varpi_{n}+\eta {\left(\lambda_{n}-\phi \right)}_{n}a_{n}\\ =\varpi_{n}+\eta \varsigma_{n}a_{n}. \end{array}$$

The relationship between the gradient vector, the cost function, the and dynamic vector factor *η*_*t*_:

(18) $$\begin{array}{c} \varpi_{n+1}=\varpi_{n}+\Delta \varpi_{n}\\ =\varpi_{n}-\eta \nabla P\left(\varpi_{n}\right)+\eta_{t}\left(\varpi_{n}-\varpi_{n-1}\right). \end{array}$$

Because *ϖ*_*n*_ − *ϖ*_*n*−1_=Δ*ϖ*_*n*−1_, formula (18) can be transformed into

(19) $$\begin{array}{c} \varpi_{n+1}=\varpi_{n}+\Delta \varpi_{n}\\ =\varpi_{n}-\eta \nabla P\left(\varpi_{n}\right)+\eta_{t}\left[-\eta \nabla P\left(\varpi_{n-1}\right)\right]. \end{array}$$

Compare the non-incremental and incremental cases, respectively, and test the performance of the incremental decision tree algorithm, the ID3 algorithm, and the Bayesian algorithm. Using this dataset, non-incremental learning is performed by the incremental decision tree algorithm, the ID3 algorithm, and the Bayesian algorithm. The time-consuming situation of the three algorithms for non-incremental learning is shown in Figure 7.

RETRACTED

It can be seen from Figure 7 that the incremental decision tree algorithm is generally more time-consuming in terms of learning time, which is also an inevitable result. The accuracy of the three algorithms for non-incremental learning is shown in Figure 8.

It can be concluded from Figure 8 that the classification accuracy of the incremental decision tree algorithm is 3.75% higher than that of the ID3 algorithm. Compared with the Bayesian algorithm, this algorithm improves the classification accuracy by 8.64%. Therefore, the classification accuracy of the incremental decision tree algorithm is better than the two algorithms.

Using this dataset, incremental learning is performed by the incremental decision tree algorithm and the ID3 algorithm, respectively. The time-consuming situation of incremental learning for the two algorithms is shown in Figure 9.

The incremental decision tree algorithm and the ID3 algorithm perform incremental learning, and the accuracy of the two algorithms for incremental learning is shown in Figure 10.

It can be concluded from Figure 10 that the classification accuracy of the algorithm in this paper is 2.64% higher than that of the ID3 algorithm. Based on it, it can be concluded that the actual classification accuracy of the incremental decision tree algorithm in this paper is significantly better than the Bayesian algorithm and the ID3 algorithm, and it can meet the requirements of incremental learning. The disadvantage is that it takes extra time to sell, which is understandable. In general, it can handle the inadequacy of the decision tree algorithm for incremental learning and achieve the expected goal.

RETRACTED

## 4. Discussion

Cluster analysis is an unsupervised learning algorithm that clusters data into clusters based on similarity. Cluster analysis is different from the data classification method. Data classification is to determine the boundary of a specific category based on the existing expert knowledge, and then classify the data according to this boundary. The cluster analysis does not know the clear definition of the category in advance. It mainly estimates the degree of similarity between the data based on the similarity measure defined by the clustering algorithm, finds out the groups of data with higher similarity, and aggregates them into clusters, i.e., produces the desired clustering results. If one wants to use the clustering algorithm to obtain useful knowledge, the operator needs to have an in-depth understanding of the analysis data and related domain knowledge to more accurately evaluate the accuracy of the clustering results.

Cluster analysis can play its role in clustering at any step in the complete knowledge discovery process and get the corresponding processing results. For example, in the process of data preprocessing, the results of the preprocessing can be easily obtained for data with a relatively simple structure and stored in the data warehouse. For data with a relatively complex structure and relatively closely related data, it is difficult to obtain the expected results through simple analysis and processing, and hence cluster analysis can be used. It obtains the association relationship between the data to grasp the data as a whole and obtain a better preprocessing effect.

Association rules can not only be used to analyze the association model between products, but also to recommend products to customers to improve cross-selling capabilities. The discovery of association rules can be done offline. As the number of commodities increases, the number of rules increases exponentially. However, through the decision-maker's choice of support and confidence, the selection of interested modes and algorithms, the efficiency can also be improved.

## 5. Conclusion

In the actual application process, since the data sample set will not be collected at the beginning, more and more data will be generated over time. In other words, in practical applications, the incremental problem is almost certainly an important problem to be encountered. This article first briefly introduces the research status of data mining and then gives a detailed description of data warehouse and data mining technology, including definitions, characteristics, and architecture. Secondly, this article introduces the design of an economic intelligent system, including the design environment and the specific implementation process of the system. Finally, this paper proposes an incremental decision tree algorithm and tests the dataset, and the result meets the expected goal. There are many data mining methods, and this article only discusses two preliminarily. In future work, how to further study more optimized and efficient algorithms based on actual work, and apply the improved algorithms to economic intelligence systems are all issues worthy of further discussion.

RETRACTED

## Figures and Tables

**Figure 1:** Data warehouse architecture.

**Figure 2:** Basic framework of a metadata management system.

**Figure 3:** OLAP engine technology framework diagram.

**Figure 4:** Three-level structure of a DM system.

**Figure 5:** OLAP modeling basic framework diagram.

**Figure 6:** OLAP analysis service module's basic framework diagram.

**Figure 7:** Time consumption of the three algorithms for non-incremental learning.

**Figure 8:** Accuracy of the three algorithms for non-incremental learning.

**Figure 9:** Time consumption of the two algorithms.

**Figure 10:** Accuracy of the two algorithms for incremental learning.

**Table 1:** Difference between online analysis processing and online thing processing.

	OLTP	OLAP
User	Operators, bottom management	Decision makers, senior management
Function	Daily operation handling	Analytical decision making
DB design	Application-oriented	Theme-oriented
Number of users	Thousands	Hundreds
Work unit	Simple services	Complex queries
Access	Read and write dozens of records	Read tens of thousands of records
DB size	100MB-GB	100GB-TB
Data	Current, up-to-date, detailed, two-dimensional, discrete	Historical, aggregated, multidimensional, integrated, unified

**Table 2:** Example of association rules.

Transaction ID	Purchase of goods	Frequent item set	Support level (%)
2000	*A*, *B*, *C*	{*A*}	75
1000	*A*, *C*	{*B*}	50
4000	*A*, *D*	{*C*}	50
5000	*B*, *E*, *F*	{*A*, *C*}	50

**Table 3:** Development environment of the economic intelligence system.

System development tools	NET-integrated development platform
Servers	Windows server 2016
Database	MySQL
System hardware standards	CPUs above PIII/IG
Memory	>16G
Operating system	Windows 10
Data warehouse creation tool	Enterprise manager

## Data Availability

Data sharing is not applicable to this article as no datasets were generated or analyzed during the current study.
